This article has been retracted.

# Construction and Application of MALDI-TOF Mass Spectrometry for the Detection of Haemophilus parasuis

**DOI:** 10.1155/2021/5588855

**Published:** 2021-04-15

**Authors:** Xiaoxu Wang, Feng Xu, Kun Ning, Liping Shen, Xinyong Qi, Jian Wang

**Affiliations:** ^1^Shanghai Animal Disease Control Center, 855 Hongjin Road, Shanghai 201103, China; ^2^Tianjin University of Traditional Chinese Medicine, Tianjin 301617, China

## Abstract

To construct a protein fingerprint database of *Haemophilus parasuis* (*H. parasuis*), thus improving its clinical diagnosis efficiency. A total of 15 *H. parasuis* standard strains were collected to establish a protein fingerprint database of *H. parasuis* using matrix-assisted laser desorption ionization time-of-flight mass spectrometry (MALDI-TOF MS), and the effects of different culture media and culture time on the quality and identification results of the protein fingerprint were investigated. The results showed that tryptone soy agar (TSA) and tryptone soy broth (TSB) media and different incubation times had no significant effect on the characteristic peaks of the protein profiles. In addition, 18 clinical isolates were used to compare the identification results of the self-built protein fingerprint database, PCR detection, and basic database. Only one strain was identified in the original VITEK-MS system database, while the self-made protein fingerprint database of *H. parasuis* was 100% accurate for the detection of 18 clinical isolate strains. The protein fingerprint database of *H. parasuis* built by our laboratory is suitable for rapid clinical diagnosis of *H. parasuis*, due to its high accuracy, efficiency, and strong specificity.

## 1. Introduction

With the improvement of the Chinese economy, the pig industry has reached a great development, so how to produce commercial pigs in a healthy and efficient way has become the key. *Haemophilus parasuis* (*H. parasuis*) disease, also known as Glässer's disease [1], is induced by *H. parasuis*, leading to the increase of body temperature, joint swelling, dyspnea, polyserositis, and arthritis in pigs [2]. It is an infectious disease with a high mortality rate, seriously endangering the health of piglets and young pigs. *H. parasuis* has brought great economic losses to the pig industry and seriously threatened the healthy development of this industry worldwide. *H. parasuis* is a Gram-negative, nonmotile, small, pleomorphic bacterium belonging to genus *Haemophilus* in the family *Pasteurellaceae* [3]. However, because it is different from other genera in this family, Dickerman et al. [4] suggested renaming *H. parasuis* to *Glasserella parasuis* (this article continues to use *H. parasuis*). The virulence varies considerably between serotypes. Virulent strains can particularly as secondary microorganism of pneumonia cause septicemia without polyserositis or Glässer's disease characterized by polyserositis, pericarditis, arthritis, and meningitis [5].

Currently, detection methods for *H. parasuis* disease include etiological detection, serological detection [6], molecular biological detection [7], and loop-mediated isothermal amplification [8]. Traditional etiological diagnosis needs pathogen isolation and culture, biochemical identification, serological or molecular biological identification, etc. However, *H. parasuis* grows slowly on the culture medium with high nutritional requirements [9]. Meanwhile, the clinical pathogen isolation and culture are often easily interfered by other miscellaneous bacteria. In general, etiological detection is difficult and time-consuming in clinical. Serological detection, with complex operation, can only detect whether pigs have been infected with *H. parasuis* but cannot be used as a basis for diagnosis of the disease. Molecular biological detection requires complicated steps including template extraction, amplification, and sequencing. Therefore, further rapid and accurate diagnosis of *H. parasuis* disease has become the primary problem.

Matrix-assisted laser desorption ionization time-of-flight mass spectrometry (MALDI-TOF MS) is a new soft ionization biomass spectrometry technology developed in recent years. It is a technology that through laser excitation of small molecular proteins or polypeptides contained in microorganisms, peptide mass fingerprints are formed and then compared with the standard fingerprints of known microorganisms in databases so as to rapidly identify microorganisms [10, 11]. MALDI-TOF MS has played a significant role in clinical [12], microbiological laboratory [13]. Compared with traditional serological and molecular biological diagnostic methods, MALDI-TOF MS is simple, rapid, accurate, economical, and with good reproducibility and high-throughput automation [14–16].

In this study, 15 serotypes of *H. parasuis* standard strains were used to construct a protein fingerprint database of *H. parasuis* using MALDI-TOF MS, so as to explore the influence of different detection conditions on identification results. In addition, 18 clinical isolates were used to compare the identification results of the self-built protein fingerprint database, PCR detection, biochemical detection, and basic database, in order to explore the application of MALDI-TOF MS technology in rapid diagnosis and identification of *H. parasuis* in veterinary clinic.

## 2. Materials and Methods

### 2.1. Strains and Sources

*Escherichia coli* standard strain ATCC 8739 was provided by BioMerieux, Inc. (France). Fifteen serotype standard strains of *H. parasuis* were purchased from the China Institute of Veterinary Drug Control. Eighteen clinical *H. parasuis* strains were isolated and preserved by Shanghai Animal Disease Control Center. The names and sources of all strains are shown in Table 1.

### 2.2. Isolation and Culture of H. parasuis

The strains were dipped with an inoculation loop under aseptic conditions and then were inoculated streaked on a chocolate plate containing 10 mg/mL NAD (Shanghai Regal Biology Technology Co., Ltd., China) and cultured at 37°C for 48 hours. The suspicious colonies were selected for gram staining and inoculated on a tryptone soy agar (TSA, Becton Dickinson and Company, USA) plate containing 5% calf serum (Thermo Fisher Scientific, USA) and 10 mg/mL NAD for culture.

Under aseptic conditions, the bacterial colonies after culture were inoculated and horizontally streaked on a sheep blood plate without NAD. Then, S*taphylococcus aureus* was selected and inoculated perpendicular to the horizontal lines. After culturing at 37°C for 24 to 48 hours, the growth of bacterial colonies was observed.

### 2.3. Biochemical Index Determination and PCR Identification of Bacteria

The suspicious colonies were selected and inoculated into glucose, lactose, galactose, mannitol, and xylose microbiochemical identification tubes, respectively. Each tube was cultured at 37°C for 24 hours at the final concentration of NAD of 10 *μ*g/mL.

The primers of *H. parasuis* (Table 2) were used for multiplex PCR amplification. The reaction system of *H. parasuis* was as follows: premix 12.5 *μ*L, DEPC water 8 *μ*L, mixed primer 3 *μ*L, and template 1.5 *μ*L. The reaction conditions were as follows: 95°C for 2 min, 94°C for 30 s, 58°C for 1 min, 72°C for 1.5 min, 29 cycles of amplification; extension at 72°C for 10 min.

### 2.4. Culture of H. parasuis in Different Culture Media

*H. parasuis* standard strain CVCC3892 was inoculated into TSA and tryptone soy broth (TSB), respectively, and cultured at 37°C for 48 hours. The bacteria growing in the two media were directly smeared on the target plate, covered with 1 *μ*L *α*-cyano-4-hydroxycinnamic acid (CHCA, BioMerieux, Inc., France) matrix solution. After completely air-dried, VITEK Mass Spectrometry (VITEK-MS, BioMerieux, France) was used to obtain the MS of the bacteria.

### 2.5. Culture of H. parasuis for Different Culture Time

*H. parasuis* standard strain CVCC3892 was inoculated into TSA and cultured in an incubator at 37°C for 24 hours or 48 hours. The single colony of the bacteria at the two time points was directly smeared on the target plate, covered with 1 *μ*L CHCA matrix solution. After completely air-dried, the MS of the strains was obtained using VITEK-MS.

### 2.6. Self-Built Protein Fingerprint Database of H. parasuis

Fifteen standard strains of *H. parasuis* were inoculated with TSA and cultured at 37°C for 48 hours. A small number of single colonies were dipped with an inoculation loop, evenly smeared on the target plate, then added with 1 *μ*L CHCA matrix solution after making double wells for each strain. The target plate was put into the machine for detection after the matrix solution was completely dried. A protein fingerprint database was constructed in line with the establishment process of VITEK MS RUO [17].

### 2.7. Verification of the Self-Built Protein Fingerprint Database by Clinical Strains

Eighteen *H. parasuis* clinical strains were inoculated into TSA, cultured at 37°C for 48 hours. The standard strain of *Actinobacillus pleuropneumoniae* (CVCC2661602) and *Pasteurella multocida* (ATCC12948) was inoculated into Columbia blood plate, cultured at 37°C for 24 hours. A small number of single colonies were taken using inoculation loop, respectively, evenly smeared on the target plate, then added with 1 *μ*L CHCA matrix solution. Finally, the target plate was put into the machine for detection after the matrix solution was completely dried. The operation was performed according to the identification process of VITEK MS RUO.

## 3. Results

### 3.1. Effect of Different Media on Protein Mass Spectra

The mass spectra of *H. parasuis* standard strain CVCC3892 inoculated in TSA and TSB media were compared. The result showed no significant difference in the characteristic peaks between the two (Figure 1), indicating that the culture medium had no significant effect on the characteristic peaks of the protein mass spectra.

### 3.2. Effect of Different Culture Time on Protein Mass Spectra

The mass spectra of *H. parasuis* standard strain CVCC3892 inoculated in TSA for 24 h and 48 h were compared. The result showed no significant difference in the characteristic peaks between the two (Figure 2).

### 3.3. Construction of Protein Fingerprint Database of 15 Standard Strains

According to the establishment process of VITEK MS RUO [17], protein mass spectra of 15 standard strains of *H. parasuis* were obtained. Forty characteristic protein peaks were ultimately retained, with at least 80% strains of each mass peak possessed 40 characteristic peaks (Figures 3(a)–3(c)). The weight of peaks was determined in accordance with the number of matches (horizontal rows) and the number of reserved characteristic peaks (vertical rows). In this study, the matching number of non-database-building bacteria was 18, and the characteristic peak was 40, so the weight of each peak was 33. Subsequently, all the number codes in super spectrum were changed to 33 in order to complete the establishment and activation of the self-built database.

### 3.4. Comparison of Identification Results between the Clinical Strain System Database and the Self-Built Database

The VITEK-MS original system database was used to identify 18 clinical *H. parasuis* isolates stored in the laboratory. The results showed that only one strain could be identified to genus *Pasteurella*, and the other strains could not be identified (Table 3).

Eighteen clinical strains isolated and identified in our laboratory were used to verify the mass spectral database of *H. parasuis*. Besides, *Pasteurella multocida* and *Bordetella* were applied for the verification of specificity of the mass spectral database (Table 3). The results showed that all the clinical strains could be detected, and the coincidence rate with the super mass spectrum was between 89.1% and 99.9%. All of *Pasteurella multocida*, *Actinobacillus pleuropneumoniae*, and *Bordetella* did not match with the new protein fingerprint database of *H. parasuis*, indicating that this new database was of strong heterogeneousness.

### 3.5. Comparison of Identification Efficiency between Clinical Strain System Database and Traditional Identification Methods

Eighteen clinical isolates of *H. parasuis* were all identified using the self-built protein mass spectra database, with identification accuracy of 100%. A total of 16 isolates were identified using the traditional PCR method, with an identification efficiency of 88.9%. Meanwhile, after isolation and culture of the strains, the efficiency of microscopic examination was 94.4% (Table 4).

## 4. Discussion

*H. parasuis* is an important pathogen posing severe infections in pigs. *H. parasuis* disease is concentrated in piglets in the nursing stage and is easily secondary to immune suppression diseases (such as porcine blue ear disease or porcine circovirus disease) in pigs [18, 19]. This disease causes huge economic losses to the pig industry worldwide. Therefore, a rapid and accurate identification method is of great significance for the prevention and treatment of *H. Parasuis* disease.

Previous studies have revealed that MALDI-TOF MS technology is applied to the identification of *foodborne yeasts* and *yeast-like fungi* [20], *filamentous fungi* [21], *mycobacteria* [22], *Nocardia* [23], and *Porphyromonas* [24]. Kuhnert et al. [25] used MALDI-TOF MS to identify *Pasteurellaceae* species and subspecies from 250 species in an efficient and simple way. Moreno et al.'s research [26] also used MALDI-TOF MS to identify animal *H*. *parasuis*. In addition, Yu et al. [27] identified 16 different proteins from *H. parasuis* by using MALDI-TOF MS. In our study, 15 serotypes *H. parasuis* standard strains were used to construct the protein fingerprint database of *H. parasuis* by MALDI-TOF MS, and the effects of different culture media and time on the identification results were studied. Meanwhile, 18 clinical isolates were used to compare the identification results of self-built database, PCR detection, and basic database. The results indicated that this protein fingerprint database of *H. parasuis* using the MALDI-TOF MS method was very stable, and culture media and time had no significant effect on it. Its accuracy and stability were similar to the traditional molecular biological detection method, but with faster detection speed.

In the process of the MALDI-TOF MS for detection of *H. parasuis*, TSA and TSB media were selected for the optimization of culture conditions, and *H. parasuis* was cultured for 24 h and 48 h, respectively. The results confirmed that both have no significant effect on the results of protein spectrum identification, indicating that *H. parasuis* requires a wide range of growth conditions. However, from the mass spectrum, there are slight differences in the intensity of characteristic peaks and the number and intensity of other small peaks in the mass spectrum of *H. parasuis* under different growth conditions. Studies have demonstrated that the mass spectrum after MALDI-TOF MS detection of *vibrio* cultured in different media is inconsistent [28], which was consistent with our results. This indicates that the growth condition of *H. parasuis* was less demanding and its growth state was consistent at different time points.

In the validation of MALDI-TOF MS detection for *H. parasuis*, before using the new protein fingerprint database, VITEK-MS was used to identify *H. parasuis* isolated strains after PCR. And the result showed that only one strain could be identified to genus *Pasteurella*, and the other strains could not be identified. Therefore, the new-built protein fingerprint database is necessary for routine testing, which can immensely improve the identification efficacy of *H. parasuis*.

In summary, compared with the traditional detection methods, the protein fingerprint database constructed by MALDI-TOF MS in this experiment for the detection of *H. parasuis* is easier to operate, economical, rapid, and more accurate. Therefore, it can be used as an effective tool for the detection of *H. parasuis*.

## Figures and Tables

**Figure 1:** Comparison of protein mass spectra of *Haemophilus parasuis* in different media.

**Figure 2:** Comparison of protein mass spectra of *Haemophilus parasuis* for different culture time.

**Figure 3:** Characteristic peaks of protein mass spectrum of *Haemophilus parasuis* standard strains. (a) Flow chart of the establishment of protein mass spectrum database; (b) screening methods of 40 characteristic protein peaks; (c) mass spectrum of 40 characteristic peaks.

**Table 1:** Information of strains.

Standard strain number	Strain name	Supplier	Clinical strain number	Separation site	Source
ATCC8739	E. coli	BioMerieux	GONGJIANPEI	Lung	Our laboratory
CVCC2661602	A. pleuropneumoniae	IVDC	0601	Lung	Our laboratory
ATCC12948	*Pasteurella multocida*	ATCC	201705	Lung	Our laboratory
CVCC3891	H. parasuis type 1	IVDC	Pmult	Lung	Our laboratory
CVCC3892	H. parasuis type 2	IVDC	C07-020	Nasal swab	Our laboratory
CVCC3893	H. parasuis type 3	IVDC	C07-019	Nasal swab	Our laboratory
CVCC3894	H. parasuis type 4	IVDC	C07-016	Nasal swab	Our laboratory
CVCC3895	H. parasuis type 5	IVDC	C07-015	Nasal swab	Our laboratory
CVCC3896	H. parasuis type 6	IVDC	C07-014	Nasal swab	Our laboratory
CVCC3897	H. parasuis type 7	IVDC	C07-013	Nasal swab	Our laboratory
CVCC3898	H. parasuis type 8	IVDC	C07-012	Nasal swab	Our laboratory
CVCC3899	H. parasuis type 9	IVDC	C07-011	Nasal swab	Our laboratory
CVCC3900	H. parasuis type 10	IVDC	C07-010	Nasal swab	Our laboratory
CVCC3901	H. parasuis type 11	IVDC	C07-009	Nasal swab	Our laboratory
CVCC3902	H. parasuis type 12	IVDC	C07-008	Nasal swab	Our laboratory
CVCC3903	H. parasuis type 13	IVDC	C07-007	Nasal swab	Our laboratory
CVCC3904	H. parasuis type 14	IVDC	C07-006	Nasal swab	Our laboratory
CVCC3905	H. parasuis type 15	IVDC	C07-005	Nasal swab	Our laboratory

Notes: all strains were isolated and preserved in our laboratory. Abbreviations: E. coli: *Escherichia coli*; IVDC: China Institute of Veterinary Drug Control; ATCC: American Type Culture Collection; H. parasuis: *Haemophilus parasui*s; A. pleuropneumoniae: *Actinobacillus pleuropneumoniae*.

**Table 2:** Primers of *Haemophilus parasuis.*

Serotype	Primer sequence		Section size (bp)
1	F	CTGTGTATAATCTATCCCCGATCATCAGC	180
	R	GTCCAACAGAATTTGGACCAATTCCTG	
2	F	CTAACAAGTTAGGTATGGAGGGTTTTGGTG	295
	R	GGCACTGAATAAGGGATAATTGTACTG	
3	F	CATGGTGTTTATCCTGACTTGGCTGT	650
	R	TCCACATGAGGCCGCTTCTAATATACT	
4	F	GGTTAAGAGGTAGAGCTAAGAATAGAGG	320
	R	CTTTCCACAACAGCTCTAGAAACC	
5/12	F	CCACTGGATAGAGAGTGGCAGG	450
	R	CCATACATCTGAATTCCTAAGC	
6	F	GATTCTGATGATTTTTGGCTGACGGAACG	360
	R	CCTATTCTGTCTATAAGCATAGACAGGAC	
7	F	CTCCGATTTCATCTTTTCTATGTGG	490
	R	CGATAAACCATAACAATTCCTGGCAC	
8	F	GGAAGGGGATTACTACTACCTGAAAG	650
	R	CTCCATAGAACCTGCTGCTTGAG	
9	F	AGCCACATCAATTTTAGCCTCATCA	710
	R	CCTTAAATAGCCTATGTCTGTACC	
10	F	GGTGACATTTATGGGCGAGTAAGTC	790
	R	GCACTGTCATCAATAACAATCTTAAGACG	
11	F	CCATCTCTTTAACTAATGGGACTG	890
	R	GGACGCCAAGGAGTATTATCAAATG	
13	F	GCTGGAGGAGTTGAAAGAGTTGTTAC	840
	R	CAATCAAATGAAACAACAGGAAGC	
14	F	GCTGGTTATGACTATTTCTTTCGCG	730
	R	GCTCCCAAGATTAAACCACAAGCAAG	
15	F	CAAGTTCGGATTGGGAGCATATATC	550
	R	CCTATATCATTTGTTGGATGTACG	
A11	F	ACAACCTGCAAGTACTTATCGGGAT	275
	R	TAGCCTCCTGTCTGATATTCCCACG	

**Table 3:** Comparison of identification results between clinical strain system database and self-built database.

Strain number	Strain name	Source	VITEK-MS original identification result	Self-built protein mass spectrum	
				Identification result	Accuracy
ATCC8739	E. coli	Merieux	E. coli	/	78.9%
CVCC2661602	A. pleuropneumoniae	IVDC	A. pleuropneumoniae	/	99.9%
ATCC12948	*Pasteurella multocida*	ATCC	Pasteurella	/	95.0%
GONGJIANPEI	H. parasuis	Isolated in laboratory	/	*Lignieresii/peuropneumoniae*	87.4%
0601	H. parasuis	Isolated in laboratory	/	*Bordetella bronchiseptica/parapertussis*	99.9%
201705	H. parasuis	Isolated in laboratory	/	*Pasteurella multocida*	99.0%
Pmult	H. parasuis	Isolated in laboratory	/	*Pasteurella multocida*	89.1%
C07-020	H. parasuis	Isolated in laboratory	/	*Pasteurella multocida*	99.9%
C07-019	H. parasuis	Isolated in laboratory	/	*H. parasuis*	99.9%
C07-016	H. parasuis	Isolated in laboratory	/	*H. parasuis*	99.9%
C07-015	H. parasuis	Isolated in laboratory	/	*H. parasuis*	99.9%
C07-014	H. parasuis	Isolated in laboratory	/	*H. parasuis*	99.9%
C07-013	H. parasuis	Isolated in laboratory	/	*H. parasuis*	99.9%
C07-012	H. parasuis	Isolated in laboratory	/	*H. parasuis*	99.9%
C07-011	H. parasuis	Isolated in laboratory	/	*H. parasuis*	99.9%
C07-010	H. parasuis	Isolated in laboratory	/	*H. parasuis*	99.9%
C07-009	H. parasuis	Isolated in laboratory	/	*H. parasuis*	99.9%
C07-008	H. parasuis	Isolated in laboratory	/	*H. parasuis*	99.9%
C07-007	H. parasuis	Isolated in laboratory	/	*H. parasuis*	99.0%
C07-006	H. parasuis	Isolated in laboratory	/	*H. parasuis*	99.9%
C07-005	H. parasuis	Isolated in laboratory	/	*H. parasuis*	99.9%

Notes: “/”: means no detection; “-”: means undetected. Abbreviations: IVDC: China Institute of Veterinary Drug Control; ATCC: American Type Culture Collection; E. coli: *Escherichia coli*; H. parasuis: *Haemophilus parasuis*; A. pleuropneumoniae: *Actinobacillus pleuropneumoniae*.

**Table 4:** Comparison of clinical strain identification efficiency.

Bacteria	Number of strain identified by self-built database (*n*)	Number of strain identified by PCR (*n*)	Number of strain identified by microscopic examination (*n*)
H. parasuis	18	16	17
Efficiency	100%	88.9%	94.4%

## Data Availability

All data generated or analyzed during this study are included in this article.
